# 18F-FDG PET/CT Image Deep Learning Predicts Colon Cancer Survival

This article has been retracted.

**DOI:** 10.1155/2023/2986379

**Published:** 2023-05-04

**Authors:** Mohan Tian, Yingci Li, Hong Chen

**Affiliations:** ^1^Center of PET/CT, Harbin Medical University Cancer Hospital, Harbin 150081, Heilongjiang, China; ^2^Department of Anesthesiology, Harbin Medical University Cancer Hospital, Harbin 150081, Heilongjiang, China

## Abstract

Colon cancer is a type of cancer that begins in the large intestine. In the process of efficacy evaluation, postoperative recurrence prediction and metastasis monitoring of colon cancer, traditional medical image analysis methods are highly dependent on the personal ability of the doctors. In the process of patient treatment, it not only increases the workload and work pressure for doctors, but also has some problems with traditional medical image analysis methods. Moreover, the traditional medical image analysis methods have problems such as insufficient prediction accuracy, slow prediction speed, and the risk of errors in prediction. When analyzing 18F-FDG PET/CT images by traditional medical image analysis methods, it is easy to cause problems such as untimely treatment plans and errors in diagnosis, which will adversely affect the survival of colon cancer patients. Although 18F-FDG PET/CT images have certain advantages in image clarity and accuracy compared with traditional medical imaging methods, the analysis method based on 18F-FDG PET/CT images also has certain effects in predicting the survival of colon cancer patients, but there are still many shortcomings: the 18F-FDG PET/CT image analysis method overly relies on the technical advantages of 8F-FDG PET/CT images; in the analysis and prediction of image data, it has not gotten rid of the dependence on the personal medical quality of the doctors; traditional medical image analysis methods are still used when analyzing and predicting images; there is no breakthrough in image analysis effects. In order to solve these problems, this paper combined deep learning theory, using three algorithms of the improved RBM algorithm, image feature extraction method based on deep learning, and regression neural network to analyze and predict 18F-FDG PET/CT images, and applied some algorithms to analyze and predict 18F-FDG PET/CT images, and also established a deep learning-based 18F-FDG PET/CT image survival analysis prediction model. Four aspects survival prediction accuracy, survival prediction speed, survival prediction precision, and physician satisfaction were studied through this model. The research results have shown that compared with traditional medical image analysis methods, the prediction accuracy of 18F-FDG PET/CT image survival analysis prediction model based on deep learning is improved by 0.83%, and the prediction speed is improved by 3.42%, as well as the prediction precision increased by 6.13%. The research results show that the deep learning-based 18F-FDG PET/CT image survival analysis prediction model established in this paper is of great significance to improve the survival rate of colon cancer patients, and also promotes the development of the medical industry.

## 1. Introduction

With the development of medical technology and imaging, 18F-FDG PET/CT detection has been applied to the diagnosis and treatment of colon cancer patients. Due to the large number of colon cancer patients, 18F-FDG PET/CT detection produces a large number of medical images, and doctors need to spend a lot of energy and time to classify and analyze these medical images, which not only reduces the efficiency of doctors, but also increases the risk of misdiagnosis. With the development of artificial intelligence and the rise of deep learning, it has become feasible to apply deep learning to the research of medical imaging to predict the survival of cancer patients. Therefore, the deep learning-based 18F-FDG PET/CT image analysis and prediction model established in this paper is feasible and of great significance.

Survival prediction analysis of colon cancer patients can improve the survival rate of patients, and many scholars have conducted research on this. Sun et al. used the machine learning method of supervised learning to study and analyze the survival data of colon cancer patients and proposed the expression characteristics of colon cancer genes [1]. Chang et al. conducted research on depressive and polypoid colon cancer tumors and found that depressive colon cancer tumors showed rapid invasive characteristics during patient survival [2]. Li et al. proposed a postoperative survival assessment method for colon cancer patients by analyzing the blood test results of colorectal cancer, combined with data classification and machine learning methods [3]. Wang et al. studied the CT images of patients with colon cancer who were admitted to the hospital and established a survival prediction model for colon cancer patients on medical imaging after observing the attenuation of colon cancer indexes by using the regression analysis algorithm [4]. Akinkuotu et al. used the colon cancer database to compare the survival rate of colon cancer patients before and after the age of 25, and found that younger colon cancer patients had a higher survival rate [5]. Parsons believed that corresponding treatment methods should be adopted for the prediction of postoperative recurrence of colon cancer patients and proposed a stratified prediction scheme based on the depth and spread of colon cancer of the patients [6]. Tian et al.'s study analyzed the informative characteristics and medical value of Calpain-9 and found that the higher the expression status of Calpain-9, the longer the overall survival of colon cancer patients [7]. Although many scholars have conducted survival prediction analysis research on colon cancer patients, there are not many studies combining 18F-FDG PET/CT images for survival prediction analysis. Therefore, this paper investigates the topic of deep learning-based 18F-FDG PET/CT images for predicting colon cancer survival.

18F-FDG PET/CT images are widely used in many studies as an imaging technique for detecting and evaluating cancer. Paul et al. used 18F-FDG PET/CT images to identify the metastasis of lung cancer and proposed a series of preventive measures in view of the possibility of lung cancer metastasis to the diaphragm and spleen [8]. Tsetsos et al. applied 18F-FDG PET/CT image technology to detect breast cancer and observe curative effect and proposed a diagnostic method for identifying whether breast cancer has lung metastasis [9]. Peng et al. constructed a diagnostic evaluation system for lymph node metastasis of nasopharyngeal carcinoma by studying 18F-FDG PET/CT images of nasopharyngeal carcinoma [10]. Ladefoged et al. conducted research on denoising of 18F-FDG PET/CT images using convolutional neural networks, resulting in a quantitative index method for determining cardiac viability in patients with heart disease [11]. Zheng et al. used 18F-FDG PET/CT and NEMA models to improve the resolution and quantitative level of diagnostic images and promoted the research and development of medical imaging [12]. Zhang et al. discussed the performance characteristics of 8F-FDG PET/CT images and used random forest regression model and other algorithms to establish an analysis and prediction model for predicting PD-L1 indicators in the study of lung adenocarcinoma [13]. Jin et al. preprocessed and locally aligned 18F-FDG PET/CT images with the Demons algorithm based on the gradient of mutual information and proposed a strategy analysis system that can accurately and quickly confirm the location of the cancer target [14]. The above studies have proved that 18F-FDG PET/CT images are widely used, but there are few studies on deep learning prediction of 18F-FDG PET/CT images.

In order to make 18F-FDG PET/CT images play a better role in the medical field and improve the accuracy of colon cancer diagnosis, the speed of diagnosis and the evaluation of the efficacy of colon cancer, postoperative monitoring, as well as to improve the survival rate of colon cancer patients, this paper combined 18F-FDG PET/CT image technology and deep learning theory to establish a deep learning-based survival analysis prediction model for 18F-FDG PET/CT images.

## 2. Prediction Model for Survival Analysis of 18F-FDG PET/CT Images Based on Deep Learning

### 2.1. Colon Cancer Image Feature Recognition and Classification System

The premise of survival analysis and prediction of 18F-FDG PET/CT images of colon cancer patients is to establish an image recognition and classification system. Classification according to the characteristics of the image can help us better perform predictive analysis work. The specific identification and classification content is shown in Figure 1.

As can be seen from Figure 1, the colon cancer image feature recognition and classification system is divided into four steps: first, the attending physician uses medical equipment to obtain 18F-FDG PET/CT images of colon cancer patients. After an initial human review of the images, some useless, repetitive images are discarded. Secondly, the image data is preprocessed, and the image data is amplified by means of data statistics and data analysis, and some irregular colon cancer image information is converted into regularly distributed digital information. Then, after defining multiple image features, the convolutional neural network model is used to identify and classify the image features. Finally, the results of the identification and classification are fed back to the doctor to facilitate the predictive analysis work.

### 2.2. Feature Extraction of 18F-FDG PET/CT Images

The quality effect of 18F-FDG PET/CT image feature extraction is directly related to the prediction effect of the survival analysis prediction model. The feature vector of an image should be based on the entire image, not just a part of the image. Moreover, the feature vectors should be distributed in a uniform state and should not be too concentrated in a certain part. Feature extraction can be divided into four parts, as shown in Figure 2.

As can be seen from Figure 2, the four parts of feature extraction are to determine the feature expression of the image, image feature analysis, storage and reanalysis, and obtain the feature extraction result. Determining the feature expression of an image refers to determining the classification type and standard of image features, which include the dimensional features, texture features, and color features of the image. The convolutional neural network can be used for analysis when determining the feature expression of the image, which makes the judgment of the classification standard of the image and the selection of the classification category more scientific and reasonable. After determining the classification standard of image features, the fully connected layer of the convolutional neural network can be used to analyze the image features. When analyzing the features of 18F-FDG PET/CT images, attention should be paid to the distinction, reliability, independence, and simplicity. Distinction refers to the feature difference value between image categories, and the difference between them should be as large as possible. Reliability means that the feature selection of the same image category should be similar, and the same object attribute cannot be judged by the criterion that is too different. Independence means that the acquisition of each image feature should be independent, and one feature value should not be used to arbitrarily infer another feature value. Simplification mainly means that the number of vector dimensions of features should be controlled within a reasonable range. Storage and reanalysis are to store the analyzed image feature value data in the image database, and then the previous data are used to detect and reanalyze the current feature value data, and finally the 18F-FDG PET/CT image feature extraction results are obtained.

### 2.3. Architecture of Survival Analysis Prediction Model

The construction of the survival analysis prediction model can provide reference opinions for the clinical diagnosis of colon cancer patients and can reduce the time spent by doctors on the selection of treatment options. It can improve the diagnostic efficiency and play an important role in predicting the survival of colon cancer patients. The 18F-FDG PET/CT image analysis and prediction model established in this paper based on deep learning theory is divided into three parts, as shown in Figure 3.

As can be seen from Figure 3, the three parts of the 18F-FDG PET/CT image analysis and prediction model are image data preprocessing, image informatization, and image feature analysis and prediction. The operation flow of image data preprocessing is to take 18F-FDG PET/CT images, screen images, and select samples. The purpose of image data preprocessing is to provide sample data for the digitized part of the image, so as to facilitate the in-depth analysis of image information. Image informatization includes three steps: scanning, feature extraction, and feature information data storage. Scanning refers to the electronic information processing of the images. Attention should be paid to the resolution of the image when scanning the image because the pixel of the image electronic process is too low, which will affect the subsequent image analysis results. Feature extraction is to process and analyze the natural features and man-made feature information of the image through the convolutional neural network to generate the feature information data of the image. Image feature analysis and prediction include data preprocessing, data analysis, and survival prediction. Feature information data storage refers to storing the feature analysis results of this image in the colon cancer database to provide reference for future research. Data preprocessing refers to data preprocessing techniques. Data preprocessing refers to data cleaning and data reduction of the extracted image feature information through data preprocessing technology. Data analysis and survival prediction refers to the automatic segmentation and processing of image feature information using the convoluted neural networks and deep learning algorithms to predict and analyze the survival of colon cancer patients. Finally, the results of the survival prediction analysis are provided to the attending physician to provide a reference for the next treatment plan.

## 3. Utilization Algorithms for Survival Analysis Prediction Models

### 3.1. Improved RBM Algorithm

The RBM algorithm is a deep learning basic algorithm consisting of a visible layer and a hidden layer. In order to give full play to the effect of the prediction model of 18F-FDG PET/CT image survival analysis, this paper combined the automatic coding algorithm to improve the RBM algorithm.

Let the visible layer be *w* and the hidden layer be *u*, then the energy function is as follows:

(1) $$\begin{array}{c} I\left(y\right)=\frac{f^{-F\left(w,u\left|\kappa \right.\right)}}{H}\text{.} \end{array}$$

*H* represents the normalized convergence factor of the energy function.

The Bernoulli function of the visible layer and the hidden layer structure model is as follows:

(2) $$\begin{array}{c} F\left(w,u\left|\kappa \right.\right)=-{\sum s}_{r=1}^{q}c_{r}w_{r}-{\sum s}_{s=1}^{p}d_{s}u_{s}-{\sum s}_{s=1}^{p}{\sum s}_{r=1}^{q}v_{rs}w_{r}u_{s}\text{.} \end{array}$$

Among them, *p* and *q* are the datasets, and *v*_*rs*_ is the connection weight between the data.

If *w*_*r*_ has a certain probability distribution, given the state parameters of *w*_*r*_ and *u*_*s*_, the conditional probability of the data unit of *w*_*r*_ and *u*_*s*_ is as follows:

(3) $$\begin{array}{c} I\left(u_{s}=1\left|w;\kappa \right.\right)=\lambda \left(\sum_{s=1}^{s}v_{rs}w_{r}+c_{r}\right)\text{,} \end{array}$$

(4) $$\begin{array}{c} I\left(w_{r}=1\left|u;\kappa \right.\right)=\lambda \left(\sum_{s=1}^{s}v_{rs}u_{s}+d_{s}\right)\text{.} \end{array}$$

Formulas (3) and (4) only express the two-layer structure of the RBM model, and the expression of the multilayer structure model is as follows:

(5) $$\begin{array}{c} F\left(w,u\left|\kappa \right.\right)=-\frac{1}{2}{\sum s}_{r=1}^{q}{\left(w_{r}-c_{r}\right)}^{2}-\sum_{s=1}^{p}d_{s}u_{s}-\sum_{s=1}^{p}\sum_{r=1}^{q}v_{rs}w_{r}u_{s}\text{.} \end{array}$$

### 3.2. Image Feature Extraction Method Based on Deep Learning

Image feature extraction refers to the use of computer technology to analyze the points of the image to determine whether the points of the image belong to an image feature. In the survival analysis of 18F-FDG PET/CT images based on deep learning, the extraction of the information features of the images is the premise and key to the survival prediction analysis.

One-dimensional signal of image classification feature vector is as follows:

(6) $$\begin{array}{c} e\left(s\right)=\underset{j}{\sum }d_{i+1},j\vartheta_{i+1},j\text{.} \end{array}$$

If *U*_*i*+1_=*U*_*i*_+*V*_*i*_, the one-dimensional signal can be described as follows:

(7) $$\begin{array}{c} e\left(s\right)=\underset{c}{\sum }d_{ic}\vartheta_{ic}\left(s\right)+\underset{c}{\sum }f_{ic}\gamma_{ic}\left(s\right)\text{.} \end{array}$$

Among them, *U*_*i*+1_ is the subspace of the one-dimensional signal, *d*_*ic*_ and *f*_*ic*_ represent the scale coefficient and wavelet coefficient, respectively, and $\underset{c}{\sum }d_{ic}\vartheta_{ic}\left(s\right)$ and $\underset{c}{\sum }f_{ic}\gamma_{ic}\left(s\right)$ refer to the low frequency and high frequency of the one-dimensional signal.

The calculation formulas of scale coefficient and wavelet coefficient are as follows:

(8) $$\begin{array}{c} d_{ic}=\underset{j}{\sum }l_{0\left(j-2c\right)}\left(s\right)d_{i+1,j}\text{,} \end{array}$$

(9) $$\begin{array}{c} f_{ic}=\underset{j}{\sum }l_{1\left(j-2c\right)}\left(s\right)f_{i+1,j}\text{.} \end{array}$$

The two-dimensional scale function of the 18F-FDG PET/CT image is as follows:

(10) $$\begin{array}{c} \vartheta \left(a,b\right)=\vartheta \left(a\right)\vartheta \left(b\right)\text{.} \end{array}$$

Among them, *f*(*a*, *b*) represents the two-dimensional signal of the 18F-FDG PET/CT image.

Orthogonal basis function of 18F-FDG PET/CT image after wavelet transformation is as follows:

(11) $$\begin{array}{c} M_{1}f\left(a,b\right)\left\{\begin{array}{c} \lambda^{1}\left(a,b\right)=\vartheta \left(a\right)\lambda \left(b\right)\\ \lambda^{2}\left(a,b\right)=\lambda \left(a\right)\vartheta \left(b\right)\\ \lambda^{3}\left(a,b\right)=\lambda \left(a\right)\lambda \left(b\right) \end{array}\right)\text{.} \end{array}$$

After further analysis of 18F-FDG PET/CT images, it can be obtained as follows:

(12) $$\begin{array}{c} B_{1}f\left(a,b\right)=\langle f\left(a,b\right),2^{-q}\vartheta \left(2^{-p}a-h_{1}\right)\vartheta \left(2^{-q}a-h_{1}\right)\rangle \text{,} \end{array}$$

(13) $$\begin{array}{c} E_{1}f\left(a,b\right)=\langle f\left(a,b\right),2^{-q}\vartheta \left(2^{-p}a-h_{1}\right)\lambda \left(2^{-q}a-h_{1}\right)\rangle \text{,} \end{array}$$

(14) $$\begin{array}{c} M_{1}f\left(a,b\right)=\langle f\left(a,b\right),2^{-q}\lambda \left(2^{-p}a-h_{1}\right)\vartheta \left(2^{-q}a-h_{1}\right)\rangle \text{,} \end{array}$$

(15) $$\begin{array}{c} N_{1}f\left(a,b\right)=\langle f\left(a,b\right),2^{-q}\lambda \left(2^{-p}a-h_{1}\right)\lambda \left(2^{-q}a-h_{1}\right)\rangle \text{.} \end{array}$$

Among them, *B*_1_*f*(*a*, *b*) is the low-frequency subimage of the 18F-FDG PET/CT image feature, *E*_1_*f*(*a*, *b*) is the detail feature information subimage in the horizontal direction of the image, *M*_1_*f*(*a*, *b*) is the vertical detail feature subimage, and *N*_1_*f*(*a*, *b*) is the diagonal detail feature subimage of the image.

### 3.3. Recurrent Neural Network

Recurrent neural network, as a deep learning algorithm, can play an important role in the recognition, classification, and analysis of information features of 18F-FDG PET/CT images.

Set the input vector of the regression neural network as *H* and the output vector as *L*, the regression result is as follows:

(16) $$\begin{array}{c} \hat{L}=G\left(l/H\right)=\frac{\int_{-\infty }^{\infty }lf\left(H,l\right)el}{\int_{-\infty }^{\infty }f\left(H,l\right)el}\text{.} \end{array}$$

*f*(*h*, *l*) is the joint probability density of the output vector and the input vector.

If the set of each 18F-FDG PET/CT image sample by *j* is {*h*_*p*_, *l*_*q*_}_*p*=1_^*j*^, there are

(17) $$\begin{array}{c} \hat{f}\left(H,l\right)=\frac{1}{j\left(2\pi \right)\kappa +1/2\alpha^{\kappa +1}}\overset{j}{\underset{p=1}{\sum }}\exp\left[-\frac{{\left(H-H_{p}\right)}^{S}\left(H-H_{p}\right)}{2\alpha^{2}}\right]•\;\exp\;\left[-\frac{{\left(H-L_{P}\right)}^{2}}{2\alpha^{2}}\right]\text{.} \end{array}$$

Among them, $\hat{f}\left(H,l\right)$ is the density function of the image set, and *κ* is the feature dimension of the image.

The formula for calculating $\hat{L}\left(H\right)$ is as follows:

(18) $$\begin{array}{c} \hat{L}\left(H\right)=\frac{\sum_{p=1}^{j}\left[-{\left(H-H_{p}\right)}^{S}\left(H-H_{p}\right)/2\alpha^{2}\right]\int_{-\infty }^{+\infty }l\;\exp\;\left[-{\left(L-L_{P}\right)}^{2}/2\alpha^{2}\right]el}{\sum_{p=1}^{j}\left[-{\left(H-H_{p}\right)}^{S}\left(H-H_{p}\right)/2\alpha^{2}\right]\int_{-\infty }^{+\infty }\exp\;\left[-{\left(L-L_{P}\right)}^{2}/2\alpha^{2}\right]el}\text{.} \end{array}$$

According to the relevant calculation, it can be obtained as follows:

(19) $$\begin{array}{c} \int_{-\infty }^{+\infty }ym^{-y^{2}}ey=0\text{.} \end{array}$$

Formula (18) can be transformed into the following:

(20) $$\begin{array}{c} \hat{L}\left(H\right)=\frac{\sum_{p=1}^{j}L_{P}\exp\;\left[-{\left(H-H_{p}\right)}^{S}\left(H-H_{p}\right)/2\alpha^{2}\right]}{\sum_{p=1}^{j}\exp\;\left[-{\left(H-H_{p}\right)}^{S}\left(H-H_{p}\right)/2\alpha^{2}\right]}\text{.} \end{array}$$

Among them, $\hat{L}\left(H\right)$ represents the regression result of the output vector *L* with respect to the input vector H=(*h*_1_, *h*_2_, ..., *h*_*j*_), *L*=(*l*_1_, *l*_2_, ..., *l*_*p*_).

## 4. Meta-Analysis of Colon Cancer Survival Prediction

Although there are many studies on colon cancer survival prediction, some studies lack systematic discussion, and the conclusions of the article lack quantitative analysis [15]. Therefore, this paper makes a meta-analysis of colon cancer survival prediction research.

In this paper, the two keywords “colon cancer” and “survival prediction” were searched in academic journal database and Wanfang database by means of literature search. After the inclusion criteria of the literature were determined, 5 high-quality literature were selected, as shown in Table 1.

According to the inclusion criteria, the 5 selected literature were summarized, and the prediction scheme of the survival rate of colon cancer patients was analyzed. The heterogeneity test showed good homogeneity among the studies.

In this paper, meta-analysis of the 5 included literatures was carried out, which could systematically and objectively carry out a comprehensive evaluation of the survival prediction of colon cancer patients. It can quantitatively analyze the research results and has an important enlightenment effect on the 18F-FDG PET/CT image survival analysis prediction model studied in this paper. Although the literature selected in this paper is not enough and the analysis is not enough, the meta-analysis shows that providing a survival analysis prediction scheme is effective in improving the survival rate of colon cancer patients.

## 5. 18F-FDG PET/CT Image Analysis to Predict Colon Cancer Survival Experimental Design

This paper selected 50 colon cancer patients from two hospitals and divided them into two groups of 25 people each. One group used the deep learning-based 18FCT image survival analysis prediction model to predict the survival of patients, which is called the experimental group in this paper; another group used traditional medical image analysis methods to perform survival prediction analysis based on the patients' 18FCT images and was called the control group. Through a 12-month experimental test on the four aspects of prediction accuracy, prediction speed, prediction precision, and doctor's satisfaction of the two survival prediction methods, the experimental results were obtained and analyzed.

## 6. 18F-FDG PET/CT Image Analysis to Predict the Experimental Results of Colon Cancer Survival

### 6.1. The Accuracy of Survival Prediction

When performing survival prediction analysis on 18F-FDG PET/CT images of colon cancer patients, if the predicted result is larger than the actual result, the treatment and maintenance plan taken by the doctor must be more radical than the original one. If the predicted result is smaller than the actual result, the doctor will adopt a relatively conservative treatment and maintenance plan. Whether it is too aggressive or too conservative treatment and maintenance plan, it is not conducive to the postoperative recovery of colon cancer patients. 10 survival analysis predictions were performed for each colon cancer patient every month, and the average of the prediction accuracy results for each person in 12 months was used as the data source. The specific content is shown in Figure 4.

Overall, the prediction accuracy of the experimental group was higher than that of the control group, indicating that using the deep learning-based 18F-FDG PET/CT image survival analysis prediction model is better than using the traditional medical image analysis method, and the prediction accuracy is improved, which is beneficial to the postoperative treatment and condition monitoring of colon cancer patients. The prediction accuracy data of the experimental group were mostly above 99%, and the prediction accuracy data of the control group were mostly around 98%, indicating that the 18F-FDG PET/CT image survival analysis prediction model played a role in improving the prediction accuracy. The average accuracy of the experimental group was 99.40%, the average accuracy of the control group was 98.58%, the average accuracy of the experimental group was 0.82% higher than that of the control group, and the average accuracy of the experimental group was 0.83% higher than that of the control group. In the survival prediction analysis of colon cancer, as long as the prediction accuracy can be improved a little, it will help the survival of colon cancer patients.

### 6.2. The Speed of Survival Prediction

When performing survival prediction analysis on 18F-FDG PET/CT images of colon cancer patients, faster prediction analysis results can help doctors better understand the condition of colon cancer patients. The specific content of the predicted speed is shown in Figure 5.

As can be seen from Figure 5, compared with the control group, the prediction model of 18F-FDG PET/CT image survival analysis based on deep learning took less prediction time. The lowest prediction time of the experimental group was 22.3 minutes, while the lowest prediction time of the control group was 24.5 minutes. In terms of the highest prediction time, the prediction time of the experimental group was 46.5 minutes, and the prediction time of the control group was 47.2 minutes. The predicted time data for the control group was not as good as the experimental group, both for the highest predicted time and the lowest predicted time, which shows that the 18F-FDG PET/CT image survival analysis prediction model can not only improve the prediction speed in general analysis and prediction, but also has an optimization effect in terms of speed in the more complex analysis and prediction. The average prediction time of the experimental group was 33.924 minutes, and the average prediction time of the control group was 35.128 minutes. Compared with the control group, the average prediction time of the experimental group increased by 3.42%.

### 6.3. Precision of Survival Prediction

In this paper, multiple predictions were made in the prediction and analysis of 18F-FDG PET/CT images of colon cancer patients in order to better improve the prediction accuracy. It analyzes the precision of the forecast according to the error difference of the 12-month statistical forecast results. The specific content is shown in Figure 6.

The precision of the image predictions was expressed in terms of the error parameter, which was generally lower in the experimental group than in the control group over the 12-month study. The error parameter of the experimental group showed a downward trend. The error parameter of the first month was 5.23 and it dropped to 2.25 in the last month. The error parameter of the control group decreased in the first four months, but the change trend was not stable after that, and the error parameter of the last month was 4.26. It shows that the 18F-FDG PET/CT image survival analysis prediction model based on deep learning has stability in reducing error parameters and improving prediction precision. The average error parameter of the experimental group was 3.83, and the average error parameter of the control group was 4.08. The average prediction precision of the experimental group was 6.13% higher than that of the control group, indicating that the deep learning-based 18F-FDG PET/CT image survival analysis prediction model has a significant effect on improving the prediction accuracy.

### 6.4. Doctor Satisfaction

This article interviewed 20 attending physicians for colon cancer, 10 of whom used the deep learning-based 18F-FDG PET/CT image analysis prediction model to diagnose and predict colon cancer patients, another 10 doctors used traditional tumor imaging image diagnosis methods to analyze 18F-FDG PET/CT images for the diagnosis and survival prediction. The specific results are shown in Figure 7.

As can be seen from Figure 7, the colon cancer attending physician's evaluation of the deep learning-based 18F-FDG PET/CT image survival analysis prediction model is higher than the evaluation of the traditional tumor imaging image diagnosis method. In the experimental group, there are 3 satisfaction evaluation indicators higher than 9 points, while only one in the control group. The highest satisfaction evaluation data in the experimental group was 9.54 and the lowest was 8.47, while the highest in the control group was 9.21 and the lowest was 8.12, indicating that the 18F-FDG PET/CT image analysis prediction model is more supported and recognized by doctors. The average satisfaction evaluation index in the experimental group was 8.941, and the average satisfaction evaluation index in the control group was 8.576. Compared with the control group, the average satisfaction evaluation index in the experimental group increased by 4.08%, indicating that doctors found that the 18F-FDG PET/CT image survival analysis prediction model can improve the prediction accuracy and prediction speed. The effect of 18F-FDG PET/CT image survival analysis prediction model has been recognized by doctors.

## 7. Conclusion

In order to solve the problems that traditional medical image analysis methods have insufficient prediction accuracy, slow prediction speed, and the risk of error in prediction, and to improve the accuracy and efficiency of colon cancer survival prediction, so as to help improve the survival rate of colon cancer patients and the treatment efficiency of doctors, this paper has combined deep learning theory to study 18F-FDG PET/CT images and built a deep learning-based survival analysis prediction model for 18F-FDG PET/CT images. Experiments have proved that the deep learning-based 18F-FDG PET/CT image survival analysis prediction model can improve the accuracy of survival prediction, the speed of survival prediction, and the precision of survival prediction.

## Figures and Tables

**Figure 1:** Colon cancer image feature recognition and classification system.

**Figure 2:** Feature extraction of 18F-FDG PET/CT images.

**Figure 3:** Architecture of predictive models for survival analysis.

**Figure 4:** Accuracy of image diagnostic predictions.

**Figure 5:** Speed of image prediction.

**Figure 6:** Precision of image prediction.

**Figure 7:** Doctor satisfaction.

**Table 1:** Basic characteristics of the selected papers.

Authors	Year of publication	Tumor stages	Survival prediction schemes	Follow-up time	Forecast result
Chen [16]	2019	I, II, III, and IV	Positive lymph node odds ratio	5 years	LNR = 0 96.7%
					0 < LNR ≤ 0.15 94.7%
					0.15 < LNR ≤ 1.00 42.9%
Li [17]	2019	I, II, III, and IV	Evaluation of clinical risk scoring systems	12 years	The 1-, 3-, and 5-year survival rates were 86.2%, 51.7%, and 26.9%
Hu and Gong [18]	2020	I, II, III, and IV	IncRNAs	5 years	The area under the curve of the 1-, 3-, and 5-year ROC curves were 0.802, 0.828, and 0.771
Zhao and Cheng [19]	2021	III	Plasma albumin to fibrinogen ratio (A/F)	5 years	Overall survival rates in the high A/F group and the low A/F group were 81.6% and 50.0%
Zhou et al. [20]	2017	III	Multislice spiral CT (ce MDCT)	3 years	The 3-year DFS of the EMVI positive and negative groups were 52.8% and 81.5%

## Data Availability

The data that support the findings of this study are available from the corresponding author upon reasonable request.
